# Immunogenicity study to investigate the interchangeability among three different types of polio vaccine: A cohort study in Japan

**DOI:** 10.1097/MD.0000000000007073

**Published:** 2017-06-08

**Authors:** Satoko Ohfuji, Kazuya Ito, Motoki Ishibashi, Shizuo Shindo, Yoshio Takasaki, Takashi Yokoyama, Takato Yokoyama, Yuji Yamashita, Keigo Shibao, Takashi Nakano, Tomomi Tsuru, Shin Irie, Yoshio Hirota

**Affiliations:** a Department of Public Health, Osaka City University Graduate School of Medicine, Osaka; b PS Clinic, Medical Co. LTA; c Shindo Pediatric Clinic; d Takasaki Pediatric Clinic; e Yokoyama Pediatric Clinic; f Yamashita Pediatric Clinic; g Shibao Clinic, Fukuoka; h Department of Pediatrics, Kawasaki Medical School, Okayama; i Medical Co. LTA; j Clinical Epidemiology Research Center, Medical Co. LTA; k College of Healthcare Management, Fukuoka, Japan.

**Keywords:** immune response, infants, interchangeability, polio vaccine, safety

## Abstract

In Japan, the routine immunization program with oral polio vaccine (OPV) has been suspended since September 2012, when a program with 4 doses of inactivated monovalent polio vaccine (IPV) or quadrivalent vaccine against diphtheria, pertussis, and tetanus with IPV (DTaP-IPV) was introduced. The aim of this study was to examine the interchangeability among these 3 types of polio vaccines.

We conducted a prospective cohort study at 5 pediatric clinics in Japan. A total of 153 infants were assigned to 1 of the 4 groups by considering the vaccination history of OPV and trivalent vaccine against DTaP. Eleven infants with a history of OPV received 3 doses of DTaP-IPV; 49 infants with a history of OPV and DTaP received 3 doses of IPV; 50 polio vaccine-naïve infants received 2 doses of IPV followed by 2 doses of DTaP-IPV; and 43 polio vaccine-naive infants received 2 doses of DTaP-IPV followed by IPV. The immunogenicity after polio vaccination was evaluated among these 4 groups.

After 2 doses of polio vaccination, more than 80% of the infants exhibited a neutralization antibody titer ≥1:8 for all Sabin strains and wild strains in all groups. After the third dose, the seroprotection proportion (i.e., a neutralization antibody titer ≥1:8) reached about 100%. After the fourth dose, a neutralization antibody titer exceeded the required protective levels (i.e., a neutralization antibody titer ≥1:8) considerably in all groups.

Four doses of polio vaccines induced a sufficient level of immunity in Japanese infants, irrespective of vaccine combinations or order.

## 1 Introduction

As a preventive measure for polio in Japan, 2 doses of oral polio vaccine (OPV) had been administered to children aged 3 to 90 months since 1961. OPV is easy to administer, inexpensive, and induces optimal intestinal mucosal immunity.^[1]^ This program had led to a dramatic decline in polio cases, with no polio infections from wild strains reported in Japan since 1980.^[2]^ However, OPV is associated with rare cases of vaccine-associated paralytic poliomyelitis (VAPP). VAPP can occur in recently vaccinated individuals or in susceptible individuals indirectly exposed to vaccine virus, as can occur in close contacts of vaccinated individuals.^[3,4]^ The VAPP risk has been estimated at about 4 cases per million births.^[5]^ As no polio infection from wild strains had been reported for several decades in Japan, public concern regarding VAPP cases was increasing.^[2,4]^

Many countries that no longer experience infection with wild polio virus have transitioned to using the safer inactivated polio vaccine,^[6]^ permitting these nations to maintain herd immunity against polio while keeping VAPP risks under control.^[7]^ Based on the practice in these other countries, a program of routine immunization with 2 doses of OPV has been suspended in Japan since September 2012. As an alternative, Japan has implemented a new polio vaccination program with 4 doses (i.e., 3 doses to prime immunity and 1 booster dose) of inactivated monovalent polio vaccine (IPV) or quadrivalent vaccine against diphtheria, pertussis, and tetanus with IPV (DTaP-IPV).^[2]^

However, there have been some concerns about switching the vaccination program from OPV to IPV and DTaP-IPV. Information was needed regarding the immunogenicity and safety of IPV only and DTaP-IPV only,^[8–12]^ as well as regarding the results of administering IPV or DTaP-IPV to children who had previously received 1 dose of conventional OPV. In addition, OPV, IPV, and DTaP-IPV have different backgrounds in terms of both route of vaccination and manufacturing process. Specifically, OPV and DTaP-IPV are manufactured from Sabin-derived polio virus strains, whereas IPV is derived from wild polio virus strains.^[2]^ Thus, the Japanese government sought to address the question of the immunogenicity and safety of these vaccines in the cases of infants receiving these different types of polio vaccines in various combinations and order.

To provide information for a national decision about the polio vaccination program, the present study investigated the interchangeability among different 3 types of polio vaccine (OPV, IPV, and DTaP-IPV) in infants and young children.

## 2 Methods

### 2.1 Studied subjects

Healthy infants and children aged 3 to 74 months without any history of poliomyelitis, diphtheria, pertussis, or tetanus were enrolled between November 2011 and March 2012, at 5 pediatric clinics in Fukuoka city. The exclusion criteria were as follows: obvious history of anaphylaxis caused by food or drugs; receipt of any live vaccine within the preceding 27 days; receipt of any inactivated vaccine within the preceding 6 days; receipt of any blood transfusion or gamma globulin preparation within the preceding 3 months; receipt of immunosuppressants (except for external use), gamma globulin preparation (≥200 mg/kg), prednisolone (≥2 mg/kg/day) as an adrenocorticosteroid preparation (except for external use), or immunosuppressive therapy (including radiotherapy) within the preceding 6 months; congenital or acquired immunodeficiency; participation in a separate clinical trial (including individuals who had completed a clinical trial in the last 6 months); and individuals who pediatricians deemed ineligible to participate in this study. Parents or guardians of the participating children received an explanation of the study from their pediatrician and provided written informed consent before participation. The study protocols were approved by the Clinical Study Review Board of Medical Co. LTA and the ethics committee at the Osaka City University Graduate School of Medicine. This study was performed in accordance with the Declaration of Helsinki and was registered on UMIN-Clinical Trial Registry (UMIN000022692).

### 2.2 Study design

In this prospective cohort study, the study subjects were included in 1 of the 4 groups by considering the vaccination history of OPV and trivalent vaccine against DTaP. In order to satisfy the requirements of the routine vaccination program while participating in this study (i.e., a total of 4 doses of polio vaccine and 4 doses of DTaP vaccine), children who had received 1 dose of OPV and 1 or no doses of DTaP at the time of recruitment, regarding as Group A, received the remaining 3 doses of polio vaccination using DTaP-IPV as part of this study (Table 1). Children who had received 1 dose of OPV and 2 or more doses of DTaP at the time of recruitment (i.e., Group B) received the remaining 3 doses of polio vaccination using IPV as part of this study. Children who had no history of OPV and had received 1 or no doses of DTaP were entered onto this study from Dose 1 of polio vaccination and were assigned to Group C or Group D. Children in Group C were vaccinated first with 2 doses of DTaP-IPV and then with 2 doses of IPV, whereas those in Group D were vaccinated first with 2 doses of IPV and then with 2 doses of DTaP-IPV.

**Table 1:** Study design: combination and order of polio vaccines.

The above 4 groups were primarily configured within the limits of the total research cost. Details of this configuration are as follows. Groups A and B comprised children who had been vaccinated with OPV as Dose 1 and were due to be vaccinated with either DTaP-IPV or IPV. Ideally, vaccination between Dose 2 and 4 should have been provided as various combinations of DTaP-IPV and IPV. However, we expected that if there was some effect of crossover boosters after antibodies had been induced, then it could, to a certain extent, be predicted from the results of Groups C and D. Groups C and D were administered 2 doses of either DTaP-IPV or IPV and subsequently were administered crossover boosters. Although the effect of administering a combination of Doses 1 and 2 cannot be determined based on our data, the results of observations from Groups C and D are applicable in interpreting the results of Groups A and B. Thus, we gave priority to switching after Dose 2, as applied for Groups C and D.

### 2.3 Information collection

At the time of recruitment, the following information was obtained by means of a self-administered questionnaire completed by each child's parent or guardian: sex, date of birth, gestational age at infant's birth, birth weight, current body weight, age of each parent at infant's birth, birth order, and vaccination history (type(s) and date(s) of vaccination). To obtain accurate information on vaccination history, data were collected upon checking the maternity record book, given that (in Japan) the vaccination history is usually recorded in the maternity record book maintained by individuals.

### 2.4 Vaccines

IPV was obtained as IMOVAXPolio, manufactured by Sanofi Pasteur SA, Lyon, France, and supplied as a sterile suspension in a prefilled single-dose syringe (0.5 mL) containing inactivated wild polio virus Type 1 (Mohoney strain; 40D-antigen units), Type 2 (MEF1 strain; 8D-antigen units), and Type 3 (Saukett strain; 32D-antigen units). No adjuvant was included in IPV. DTaP-IPV was obtained as TETRABIK, manufactured by The Research Foundation for Microbial Diseases of Osaka University (BIKEN), Osaka, Japan, and supplied as a sterile suspension in a prefilled single-dose syringe (0.5 mL) containing pertussis antigen (4 units), diphtheria toxoid (23.5 units and above), tetanus toxoid (13.5 units and above), and inactivated Sabin polio virus Type 1 (LSc, 2ab strain; 1.5D-antigen units), Type 2 (P712, Ch, 2ab strain; 50D-antigen units), and Type 3 (Leon, 12a1b strain; 50D-antigen units). Aluminum-containing adjuvants were included in DTaP-IPV. The route of inoculation for both IPV and DTaP-IPV was subcutaneous; administration was not simultaneous with other vaccines.

### 2.5 Serum sampling and measurement of antibody titer

Serum samples were collected at the following 4 time points: recruitment; 4 weeks after Dose 2 (S2); 4 weeks after Dose 3 (S3); and 4 weeks after Dose 4 (S4). Recruitment corresponded to S1 for members of Groups A and B (individuals who had already received 1 dose of OPV) or S0 for members of Groups C and D (individuals who had not previously received any polio vaccine). All serum specimens were stored at –80°C until measurement. The neutralization antibody titers for Sabin strain Types 1, 2, and 3 were measured by the laboratory at the Surveillance Section, the Research Foundation for Microbial Diseases of Osaka University; while the neutralization antibody titers for wild-strain Types 1, 2, and 3 were measured by at Global Clinical Immunology, Sanofi Pasteur. All of these titer determinations were performed according to the method recommended by World Health Organization.^[13]^ Antipoliovirus types 1, 2, and 3 antibodies were measured by a neutralization assay, the poliovirus micrometabolic inhibition test, which measured the functional serum antibody response to poliovirus by utilizing Vero cells (African green monkey kidney cells) and wild-type polio virus strains 1, 2, and 3 (Mahoney, MEF-1, and Saukett, respectively), and Sabin-type polio virus strains 1, 2, and 3 (LSc, 2ab strain, P712, Ch, 2ab strain, and Leon, 12a1b strain) as the challenge virus. The Karber method was used to determine the serum dilution that neutralized 50% of the challenge virus. Results were expressed as titers (1/dilution). These assays for all 6 poliovirus strains were performed on blood samples obtained at 4 time points and all serological analyses were performed in an observer–blind manner. Antibodies associated with DTaP were not assessed as part of the present study.

### 2.6 Survey of adverse reactions

All vaccinated subjects were asked to report (through their parents or guardians completed questionnaire) selected local and systemic reactions occurring within 48 hours after vaccination. Local reactions included redness, swelling, and pain at the injection site. Systemic reactions included fever (axillary temperature ≥37.5°C), seizure, rashes, nausea, diarrhea, cough, and runny nose. In addition, serious adverse events (SAEs; those that contribute to death, are life-threatening, require hospitalization for treatment, cause permanent disability or dysfunction, or include other serious medical conditions) were collected from the participating pediatricians throughout the study. Based on the detailed information obtained for the SAEs, causality was assessed by the investigators.

### 2.7 Statistical analyses

The primary endpoint was immunogenicity. To assess the immunogenicity of polio vaccines, geometric mean titer (GMT), fold rise, and seroprotection proportion were calculated. Based on the previous immunogenicity studies of polio vaccines,^[14,15]^ seroprotection was determined as a neutralization antibody titer ≥1:8. For data processing, neutralization antibody titers <1:4 were regarded as 1:2, and reciprocal antibody titers were analyzed after logarithmic transformation. The results were converted to the original scale by calculating the antilogarithm. The significance of fold rise within a group was assessed by the Wilcoxon signed-rank test, and comparisons among the groups were made by the Kruskal–Wallis test or the χ^2^ test. The secondary endpoint was safety. To analyze descriptive information on postvaccination adverse reactions, frequencies of each local and systemic reaction were calculated. Statistical analysis for frequency comparison among the groups was conducted using the χ^2^ test. All tests were 2-sided. All analyses were performed using SAS, version 9.3 (SAS Institute).

## 3 Results

A total of 153 infants participated in this study. Among those, 11 and 49 infants were enrolled in Groups A and B, respectively, because these subjects had already received 1 dose of OPV in general vaccination program. An additional 50 and 43 polio vaccine-naive infants were enrolled in Groups C and D, respectively.

Table 2 shows the baseline characteristics of the study subjects according to study group. Infants in Groups A and B were older and had heavier current weights than those in Groups C and D, as these subjects had received OPV before 2012 (i.e., OPV use was subsequently curtailed). Other characteristics were similarly distributed among the groups. Regarding Groups A and B, median time interval from OPV was 2.5 and 2.3 months, respectively. Seroprotection proportion of Sabin-Type 1 and Sabin-Type 2 reached more than 90% at the time of recruitment, although that of Sabin-Type 3 was less than half. Similar distribution was observed in the seroprotection proportion for wild strains. Additionally, about 40% of infants in Groups C and D had antibodies against Sabin-Type 1 and Sabin-Type 2 at the time of recruitment, despite being polio vaccine-naïve. Similarly, about 10% of infants had antibodies against Sabin-Type 3 and wild strains even before polio vaccination.

**Table 2:** Baseline characteristics of infants according to the entry group^∗^.

Table 3 shows GMT and fold rise in neutralization antibody titer against polio vaccines. Since infants in Groups A and B had higher antibody titers, especially for Sabin-Type 1, Sabin-Type 2, or Wild-Type 2, at the time of recruitment (i.e., S1), the second dose of polio vaccine (whether DTaP-IPV for Group A or IPV for Group B) induced only approximately 2-fold increase in neutralization antibody titer, and the further fold rise following the third dose or fourth dose was less than 2-fold. In both Groups A and B, prevaccination (S1) titers for Type 3 were lower than those for Type 1 or 2, and thus an increase in antibody production of more than 3-fold was observed even with the fourth dose. In Groups C and D, the first 2 doses of polio vaccine induced immune responses of more than 10-fold for all strains, whether subjects were dosed with DTaP-IPV (i.e., Group C) or IPV (i.e., Group D). Although the cross-booster effect of the third dose ranged from 1.5- to 10.4-fold in Group C and from 1.1- to 2.4-fold in Group D, these fold rises with the third dose seemed to depend on the antibody titers after the second dose (S2): infants with lower antibody titers at S2 showed a higher fold rise following the third dose, whereas those with higher antibody titers at S2 showed a lower fold rise following the third dose. GMTs after the fourth dose (S4) were considerably higher than the seroprotection level in all groups, and exceeded 1:1000 for all strains other than Wild-Type 1 in Group A. Among Group A subjects (for whom all 4 doses consisted of Sabin-derived polio vaccines), the antibody titers at S4 were relatively low for Sabin-Type 3 and for all types of wild strains. Additionally, the GMT for Sabin-Type 1 was lowest in Group D, in which the first 2 doses consisted of wild strain-derived IPV and the remaining 2 doses consisted of Sabin strain-derived DTaP-IPV.

**Table 3:** Immune responses to polio vaccines according to the study group.

Table 4 shows seroprotection proportion with the polio vaccines. Regardless of vaccination combination and order, more than 80% of infants generated a neutralization antibody titer ≥1:8 for all strains after 2 doses, and the seroprotection proportion (i.e., a neutralization antibody titer ≥1:8) reached about 100% after the third dose.

**Table 4:** Seroprotection proportion to polio vaccines according to the study group.

Figure 1 shows the reported local and systemic reactions after each dose administration. All 153 subjects responded the questionnaire of adverse reactions. Redness around the injection site was reported more frequently after injection with DTaP-IPV than with IPV. Local swelling was reported at frequencies similar to those for redness. Local pain was reported by few infants, although we acknowledge that parents or guardians might not have been able to objectively distinguish infants complaining of pain. Regarding systemic reaction, fever was observed in 9% of infants in Group A, whereas fewer infants had fever after vaccination in the other groups. Diarrhea was reported in 5% to 10% of infants in each group. Cough and runny nose were reported in 10% to 20% of infants, irrespective of vaccine combination and order; these symptoms may have been unrelated to the vaccine per se, given that most vaccinations were conducted during the winter season.

**Figure 1:** Side effects after the polio vaccination according to the study group. Group A included infants who had received 1 dose of OPV; Doses 2–4 were administered using DTaP-IPV. Group B included infants who had received 1 dose of OPV; Doses 2–4 were administered using IPV. Group C included polio vaccine-naïve infants; Doses 1–2 were administered using DTaP-IPV, and Doses 3–4 were administered using IPV. Group D included polio vaccine-naïve infants; Doses 1–2 were administered using IPV, and Doses 3–4 were administered using DTaP-IPV. DTaP-IPV = quadrivalent vaccine against diphtheria, pertussis, and tetanus with IPV, IPV = inactivated monovalent polio vaccine, OPV = oral polio vaccine.

A total of 6 SAEs were reported throughout the study. In Group B, 1 infant was admitted with probable Kawasaki disease at 3 months after the third dose of IPV; a second infant was admitted with inguinal hernia at 4 months after the third dose of IPV; and a third infant was admitted with RS virus-induced pneumonia at 8 months after the third dose of IPV. In Group C, 1 infant was admitted with intussusception at 22 days after the third dose of IPV; a second infant was admitted with RS virus-induced bronchiolitis at 68 days after the third dose of IPV; and a third infant was admitted with febrile seizure at 3 months after the third dose of IPV. Notably, however, none of these SAEs appeared to be related to the polio vaccines, given that an obvious cause was determined in all cases and the time interval from vaccination to the occurrence of the respective SAE was too long to conclude a relationship to vaccination.

## 4 Discussion

The present study indicated that 4 doses of polio vaccine induced a sufficient level of immunity among Japanese infants, irrespective of vaccine combination and order. After the fourth dose, the seroprotection proportion reached about 100% for all strains, and GMTs for all strains exceeded the protective level of immunity.

Several previous studies have examined the interchangeability among different types of polio vaccines. Studies in China^[14]^ and in Guatemala^[15]^ demonstrated that IPV followed by OPV was immunogenic and noninferior to OPV only. Using infants who had received 2 previous doses of DTaP-IPV, a study in the USA demonstrated that either DTaP-IPV, OPV, or DTaP-IPV + OPV as the third dose provided a sufficient booster effect.^[16]^ Similarly, a Canadian study that targeted infants who had already received 2 doses of OPV or 3 doses of DTaP-IPV demonstrated a sufficient booster effect whether DTaP-IPV, OPV, or IPV was used for the subsequent dose.^[17]^ These results suggest the interchangeability of polio vaccines even when administered as regimens of different combinations and orders.

In the present study, however, GMTs for wild strains were relatively low in Group A, in which infants received all 4 doses of Sabin-derived polio vaccines. In addition, the GMT for Sabin-Type 1 appeared to be low in Group D, in which infants received wild-derived polio vaccine as the primary immunization. These results suggested that the type of primary immunization is important for obtaining higher immune responses to relative polio vaccine. This inference is consistent with a previous study that detected a better immune response to vaccine strains that were used as a primary dose.^[14]^ However, the results for Group C (i.e., infants who received Sabin-derived polio vaccine as the primary dose) of the present study revealed that the immune response to wild strains was as good as that to Sabin strains. Besides, the results of Group D (i.e., infants who received wild-derived polio vaccine as the primary dose) also detected similar immune responses to Sabin-Type 2 and -Type 3 strains and wild strains. Thus, although our results suggested that a better immune response was obtained for strains that were included in the primary dose, the effect of cross-boosting was adequate for the induction of appropriate antibody responses.

Regarding prevaccination titer among polio vaccine-naïve infants (i.e., Group C or Group D), about 40% of infants had the antibody for Sabin-Type 1 or Sabin-Type 2, whereas only about 10% of infants had antibodies for Sabin-Type 3 or wild strains. Thus, seroprevalence against poliovirus was high even before vaccination, consistent with the results of a previous Japanese study.^[8]^ The median age of the present study's subjects was 4 months, similar to that in the previous study.^[8]^ Additionally, high vaccination coverage (exceeding 90%) was expected among the subjects’ mothers.^[2]^ It is therefore considered that high seroprotection proportion before vaccination could be explained by the passive immunity from maternal antibodies. However, we note that a study in Cuba indicated that polio vaccine-naïve infants had a rapid decline in maternal antibodies to undetectable levels by 6 to 7 months of age.^[18]^ Taken together, these results indicate that infants should receive a primary dose of polio vaccine before 6 to 7 months of age.

As for safety, the present study showed a higher incidence of local reaction after DTaP-IPV than after IPV. It might be explained by the adjuvants and 6 antigens in DTaP-IPV. However, the reported proportion did not exceed 40%, which was a lower level than that in a previous report in Japan.^[8]^ Systemic reactions such as fever or diarrhea were reported in 5% to 10% of infants in the present study, and the proportion seemed to be similar after IPV or DTaP-IPV. The incidence of cough or nasal discharge was 10% to 20%, which was a similar level to that reported in the previous study.^[8]^ In addition, no vaccine-related SAE was reported. Thus, a regimen of 4 doses of polio vaccine was safe, irrespective of vaccine combination or order.

One strength of the present study is that all study subjects completed the study; thus, potential bias from withdrawal should not apply. However, some of the serum samples were not obtained in volumes sufficient for measuring titers against all 6 polio virus strains tested, and thus the results of antibody titer for wild strains could not be obtained for some infants. However, we note that these missing data (for antibodies against wild strains) were not related to the immune response to the strains that composed the polio vaccines. Thus, this selection bias should not affect the plausibility of the results.

The following limitations should be considered. First, the insufficient statistical power owing to the small sample size is obviously important. Particularly in Group A, small sample size might bring about unstable results. The small sample size reflected the fact that Japanese people are likely to be vaccinated according to the recommended vaccination schedule, making it difficult to find infants eligible for enrollment in Group A (i.e., subjects who had received OPV but not DTaP). Second, the present results might not sufficiently show the interchangeability among polio vaccines. The enrollment of additional groups that included several combinations and orders of polio vaccines would have yielded more meaningful results. However, we were able to identify the effect of the cross-booster at the third dose through the comparison of Group C with Group D. It is therefore expected that adequate immune responses would be obtained by using different types of polio vaccines as the second dose or the fourth dose.

## 5 Conclusion

The present study showed that 4 doses of polio vaccines induced a sufficient level of immunity and was safe in Japanese infants, irrespective of whether DTaP-IPV or IPV was followed by OPV, IPV was followed by DTaP-IPV, or DTaP-IPV was followed by IPV. To investigate the persistence of sustained immunity and timing of additional booster doses, further follow-up study of this study's subjects is ongoing.

## Acknowledgments

Sanofi Pasteur and The Research Foundation for Microbial Diseases of Osaka University are acknowledged for providing support in testing of sera.
